The article "Toward Respiratory Support of Critically Ill COVID-19 Patients Using Repurposed Kidney Hollow Fiber Membrane Dialysers to Oxygenate the Blood" was published in 2020. Journal: J Healthc Eng.

# Toward Respiratory Support of Critically Ill COVID-19 Patients Using Repurposed Kidney Hollow Fiber Membrane Dialysers to Oxygenate the Blood

**DOI:** 10.1155/2020/8862645

**Published:** 2020-11-03

**Authors:** David M. Rubin, Neil T. Stacey, Tonderayi Matambo, Claudia Do Vale, Martin J. Sussman, Tracy Snyman, Mervyn Mer, Diane Hildebrandt

**Affiliations:** ^1^Biomedical Engineering Research Group, School of Electrical and Information Engineering, University of the Witwatersrand, Johannesburg, South Africa; ^2^School of Chemical and Metallurgical Engineering, University of the Witwatersrand, Johannesburg, South Africa; ^3^Institute for the Development of Energy for African Sustainability, University of South Africa (UNISA), Florida, South Africa; ^4^Morningside Hospital, Johannesburg, South Africa; ^5^Department of Medicine, Division of Nephrology, University of the Witwatersrand, Johannesburg, South Africa; ^6^Cardio-thoracic Surgery, Milpark Hospital, Johannesburg, South Africa; ^7^Department of Chemical Pathology, University of the Witwatersrand, Johannesburg, South Africa; ^8^National Health Laboratory Service, Johannesburg, South Africa; ^9^Charlotte Maxeke Johannesburg Academic Hospital, Johannesburg, South Africa; ^10^Department of Medicine, Divisions of Critical Care and Pulmonology, University of the Witwatersrand, Johannesburg, South Africa

## Abstract

The COVID-19 pandemic has highlighted resource constraints in respiratory support. The oxygen transfer characteristics of a specific hollow fiber membrane dialyser was investigated with a view to repurposing the device as a low-cost, readily available blood oxygenator. Oxygen transfer in a low-flux hollow fiber dialyser with a polysulfone membrane was studied by passing first water and then blood through the dialyser in countercurrent to high-purity oxygen. Oxygen transfer rates of about 15% of the nominal 250 ml (STP)/min of a typical adult oxygen consumption rate were achieved for blood flow rates of 500 ml/min. Using two such dialysis devices in parallel could provide up to 30% of the nominal oxygen consumption. Specific hollow fiber dialysis devices operating with suitable pumps in a veno-venous access configuration could provide a cost-effective and readily available supplementation of respiratory support in the face of severe resource constraints.

## 1. Introduction

The COVID-19 pandemic has highlighted resource constraints in the management of respiratory distress [1], and debate continues on the merits of ventilation vs. less invasive respiratory support for COVID-19, in terms of disease management and safety of medical staff [2]. Extracorporeal membrane oxygenators (ECMOs) have been used successfully to oxygenate and decarbonate blood [3, 4], and there are a number of indications for the use of ECMO [5]. However, its use is costly and resource intensive [6].

The article "Toward Respiratory Support of Critically Ill COVID-19 Patients Using Repurposed Kidney Hollow Fiber Membrane Dialysers to Oxygenate the Blood" was published in 2020. Journal: J Healthc Eng.

Our objective is not to replace ECMO but rather to investigate repurposing of renal hollow fiber membrane dialysers (HFMDs) as cost-effective augmentation of respiratory support in resource-constrained environments.

Unlike purpose-designed ECMO membranes [7, 8], renal dialysis membranes are designed for liquid-liquid transfer of specific molecules. Nonetheless, their existing clinical approval for renal replacement therapy makes repurposing HFMDs as oxygenators an attractive option.

Nominal O_2_ consumption in adults is approximately 250 ml·min^−1^(STP) (0.357 g·min^−1^) [9]. The purpose of respiratory support is to achieve concentrations of O_2_ and CO_2_ in arterial blood that are compatible with proper organ function. Repurposed dialysers could potentially provide sufficient gas transfer to compensate for the respiratory deficit in some patients.

We investigated O_2_ transfer in a renal HFMD using water as a blood substitute. This facilitated exclusion of problems such as air bubble formation and transmembrane fluid leakage. The minimum O_2_ transfer rate in water motivated further experiments with blood.

## 2. Materials and Methods

### 2.1. Theoretical Considerations and Computational Methodology

Mass transfer in the HFMD is modelled by the following equation:

(1) $$\begin{array}{c} k_{0}A=\frac{q{\text{O}}_{2}}{LM\Delta {\text{pO}}_{2}}, \end{array}$$

where *k*_0_ is the mass transfer coefficient, *A* is the membrane area, *q*O_2_ is the rate of oxygen transferred, and *LM*ΔpO_2_is the logarithmic mean of partial pressure differences at the top and bottom of the device.

Defining the partial pressure difference between the blood inlet and the oxygen flow outlet as ΔpO_2_^top^ and between the blood outlet and oxygen flow inlet as ΔpO_2_^bottom^, and expanding the definition of logarithm mean, the expression for the product of the mass transfer coefficient and the area (*k*_*0*_*A*) becomes

(2) $$\begin{array}{c} k_{0}A=\frac{q{\text{O}}_{2}}{\left(\Delta {\text{pO}}_{2}^{\text{top}}-\Delta {\text{pO}}_{2}^{\text{bottom}}\right)/\text{ln}\left(\Delta {\text{pO}}_{2}^{\text{top}}/\Delta {\text{pO}}_{2}^{\text{bottom}}\right)}. \end{array}$$

To achieve a given *q*O_2_, this equation facilitates determination of the minimum *k*_0_*A* of the device.

As oxygen transport capacity of blood resides primarily in haemoglobin, it reaches saturation at a low partial pressure of oxygen. Thus, we can assume that oxygen transfer into blood takes place within a narrow range of partial pressures. Also, for high-purity oxygen, the *p*O_2_ may be regarded as essentially constant.

The article "Toward Respiratory Support of Critically Ill COVID-19 Patients Using Repurposed Kidney Hollow Fiber Membrane Dialysers to Oxygenate the Blood" was published in 2020. Journal: J Healthc Eng.

The oxygen-carrying capacity of blood is 8800 *μ*M of O_2_ bound to the Hb for 100% saturation [10] and dissolved O_2_ in blood is negligible. The HFMD cartridges are designed for blood flow rates up to 500 ml/min, and we evaluate oxygen-carrying capacity of blood for an Hb concentration of 15 g/100 ml and a typical oxyhaemoglobin dissociation curve.

At sea level atmospheric pressure, and for a typical venous and arterial pO_2_ of 6 and 12.7 kPa (and corresponding HbSat of 45% and 95%), respectively, the oxygen uptake in 500 ml of blood and the ΔpO_2_^top^and ΔpO_2_^bottom^are calculated and substituted into (2) to estimate the required *k*_*0*_*A*. This is repeated for an inlet venous HbSat of 25% as shown in Table 1.

It is assumed that mass transfer across the membrane is rate limiting rather than mass transfer through blood or the reaction of oxygen with haemoglobin.

### 2.2. Materials and Methods for Gas Transfer into Water

The experiments were conducted at the Biotechnology Laboratory at UNISA, Johannesburg, at an altitude of about 1700 m with atmospheric pressure about 84 kPa and temperature about 25°C.

A low-flux Leoceed-21N (Asahi Kasei Medical) hollow fiber membrane renal dialyser cartridge was used in this study. The polysulfone membrane has an effective surface area of 2.1 m^2^, and the HFMD has a priming volume of 108 ml and an internal fiber diameter and wall thickness of 185 *μ*m and 35 *μ*m, respectively. The manufacturer-specified maximum blood flow rate is 500 ml·min^−1^ (mean residence time about 13 s at this flow rate). Maximum transmembrane pressure (TMP) is rated at 80 kPa.

Tap water was deoxygenated by boiling and allowed to cool in a sealed glass bottle and measured for dissolved oxygen (SD 400 OXI L, Lovibond, Amesbury, UK). The deoxygenated water was pumped through the vertically mounted HFMD using a peristaltic pump (Qdos Chemical Metering Pumps, Watson Marlow, Cornwell, UK) via the blood inlet at 50, 200, and 500 ml·min^−1^ and discharged into a beaker covered with parafilm to minimize oxygen losses.

High-purity (>99%) oxygen (Afrox Gas, Johannesburg, South Africa) was passed countercurrent through the HFMD via the dialysate inlet, using a pressure regulator set between 60 and 80 kPa (gauge) followed by a needle valve to control flow rate at 400 ml ·min^−1^.

### 2.3. Materials and Methods for Gas Transfer into Blood

This study with human blood was approved by the Institutional Review Board of the South African National Blood Service (SANBS) Human Research Ethics Committee (certificate number: 2019/0521) and the Institutional Review Board of the University of the Witwatersrand, Johannesburg Human Research Ethics Committee (Medical) (certificate number: M200456). The experiments were conducted at the Chemical Pathology Laboratory, University of the Witwatersrand, Johannesburg, at an altitude of about 1500 m (atmospheric pressure about 85 kPa).

The article "Toward Respiratory Support of Critically Ill COVID-19 Patients Using Repurposed Kidney Hollow Fiber Membrane Dialysers to Oxygenate the Blood" was published in 2020. Journal: J Healthc Eng.

Recently expired donor whole blood (SANBS) was warmed in a water bath at 37°C and pooled in a glass flask to constitute approximately 4.5 l to which approximately 3000 units of heparin (heparin sodium mucosal, Fresenius Kabi, 5 ml of 1000·U/ml) was added.

Nitrogen sparge gas was bubbled through the blood to reduce the % oxygen saturation of haemoglobin (HbSat) to typical venous levels [11]. The nitrogen flow was gradually increased from 1 l/min until froth was visualized.

As shown in Figure 1, blood was pumped by a roller pump through the hollow fibers of a vertically mounted HFMD, from top to bottom, at 500 ml/min. The upstream placement of the roller pump reduces the risk of red blood cell lysis prior to oxygenation. Blood was discharged into a collecting flask. Oxygen was passed countercurrent at 1250 ml/min through the outside of the fibers.

The pump was placed ≈0.5 m below the base of the HFMD to achieve a pressure head, thus reducing the required suction, making sampling easier. The blood was piped through dialysis tubing fitted with inlet and outlet sampling ports (Fresenius Kabi).

After priming with normal saline, the flow was switched to blood, which was mixed by swirling, prior to and during the experiments.

Two runs were performed using a Leoceed-21N (Asahi Kasei Medical) HFMD and the third run using a Leoceed-18N (effective surface area of 1.8 m^2^ and priming volume 96 ml). A high-flux Leoceed H-type dialyser was also tested, but fluid leakage across the membrane into the gas side was noted, suggesting that this high-flux dialyser may not be suitable for oxygenation.

Two to four inlet and outlet blood samples of 1–4 ml each were taken for each run with heparin-coated syringes and analysed with a blood gas analyser (Radiometer, ABL80 FLEX CO-OX) for haemoglobin concentration (Hb), partial pressure of carbon dioxide (pCO_2_), partial pressure of oxygen (pO_2_), and haemoglobin saturation (HbSat). Bicarbonate ion concentrations (HCO_3_^−^) were calculated by the blood gas analyser.

Measurements were averaged for each run over the sample number. Measurement uncertainties were reported as ± 1 standard deviation based on rounded estimates from coefficients of variation [12, 13] and scaled for sample number.

## 3. Results

### 3.1. Experiments with Water

Oxygen was passed through the HFMD at 400 ml/min and water was run countercurrent through the inside of the hollow fibers. Inlet oxygen concentration was measured at 3.61 mg/l, at 37.1 °C

Outflow water was collected in beakers and oxygen concentration measured.  Table 2 shows these data and corresponding calculated oxygen transfer rates.

The article "Toward Respiratory Support of Critically Ill COVID-19 Patients Using Repurposed Kidney Hollow Fiber Membrane Dialysers to Oxygenate the Blood" was published in 2020. Journal: J Healthc Eng.

The low reading of 28.6 mg·l^−1^ is probably due to higher overall oxygen losses at saturation due to the slower flow rate.

Equation (2) is used to estimate *k*_0_*A* based on the minimum oxygen transfer rate of 14.6 mg·min^−1^ at 500 ml·min^−1^. Dissolved oxygen concentration is treated as negligible as haemoglobin carries most of the oxygen.

The oxygen exit stream is at atmospheric pressure, and the water inlet's partial pressure is given by the % saturation read from the dissolved oxygen meter *×* pO_2_ in air at 84 kPa, which amounts to a difference of ΔpO_2_^top^ = 72 kPa. The oxygen outlet pressure has little influence on the large driving force for mass transfer.

The ΔpO_2_^bottom^requires knowledge of the unmeasured gas pressure as it enters the HFMD. The pressure regulator reading was 60 kPa, but most of the pressure drop occurs at the needle valve. Also, prior to membrane contact, there was a contractor connection and the expansion/elbow entering the membrane unit, whereas on the discharge side there was just the expansion/elbow and a short length of tubing to the discharge. While it is not possible to exactly know the pressure in the membrane unit, it must be considerably lower than the regulator's pressure reading, and a simple estimate suggests that the relevant pressure drop is as low as 0.1 kPa.

Because the outlet water stream is at or above saturation, the partial pressure difference at that point is at most equal to that overpressure amount. Thus, the mass transfer coefficient calculations are highly sensitive to the actual pressure in this region.

For a 0.1 kPa partial pressure drop across the ΔpO_2_^bottom^ and a minimum oxygen transfer rate measured at 14.6 mg/min, equation (2) yields a *k*_0_*A* value of 1.334 mg·min^−1^·kPa^−1^. This implies a 3.4-fold larger oxygen mass transfer rate than required to fully oxygenate blood to 95% saturation for incoming pO_2_ of 45 mmHg and 1.7-fold larger than needed if the incoming pO_2_ is 25 mmHg.

Even in the unlikely case of a ΔpO_2_^bottom^of 6 kPa, the potential mass transfer rate of oxygen will be 1.4-fold larger than the minimum needed for incoming blood with oxygen partial pressure of 45 mmHg and 70% of the required amount for an incoming saturation of 25 mmHg.

### 3.2. Results for Gas Transfer in Blood

As seen in Figure 2, the dark blood entering the top and bright red blood exiting from the bottom of the HFMD is clear evidence of oxygenation.

The article "Toward Respiratory Support of Critically Ill COVID-19 Patients Using Repurposed Kidney Hollow Fiber Membrane Dialysers to Oxygenate the Blood" was published in 2020. Journal: J Healthc Eng.

Measurements from the inlet and outlet ports from two runs using a Leoceed-21N HFMD and one run using the Leoceed-18N HFMD are shown in Table 3. Samples (*n* = 2 to 4) were averaged and reported ± one standard deviation measurement uncertainty.

Measurement uncertainties for the blood gas analyser were approximated as 1% for pO_2_, pCO_2_, and Hb and 0.1% for HbSat based on the reported coefficient of variation data [12, 13]. The high values for pCO_2_ are in keeping with known changes in stored blood [14].

Oxygen content per 100 ml of blood was calculated using a conservative Hüfner constant of 1.31 as follows [15]:

(3) $$\begin{array}{c} \text{Oxygen content per 100 ml}=1.31\cdot \text{HbSat}\cdot 0.01+0.0225\cdot {\text{pO}}_{2}. \end{array}$$

Substituting the differential values for HbSat and pO_2_ between inlet and outlet into (3), the oxygen transfer rate (VO_2_) in ml(STP)·min^−1^ for a blood flow rate of 500 ml/min was calculated as shown in Table 4. This table also shows the percentage of the nominal 250 ml(STP)·min^−1^ oxygen consumption rate (VO_2,*n*_) and the % maximum (100% HbSat at the outlet at prevailing Hb) oxygen transfer rate (VO_2,max_).

Highest oxygen transfer rates were obtained on Run 1 with the 21N HFMD. Run 2 utilising the same HFMD showed diminished oxygen transfer rates compared to Run 1, probably due to fouling of the HFMD which was noted prior to the second run. Run 3 with the 18N HFMD showed the lowest oxygen transfer rates which is consistent with the smaller surface area.

Using equation (2), the product of the mass transfer coefficient and the area (*k*_0_*A*) estimates for oxygen was 0.72, 0.56, and 0.69 mg·kPa^−1^·min^−1^ for runs 1, 2, and 3, respectively. These estimates are in close agreement with theoretical *k*_0_*A* estimates for blood which ranged from 0.389 to 0.787 mg·kPa^−1^ min^−1^. These estimates are also in keeping with the minimum estimated *k*_0_*A* of 1.33 mg·kPa^−1^·min^−1^ for a minimum oxygen transfer rate of 14.6 mg·min^−1^ determined in the water experiments.

### 3.3. Mass Transfer Estimates for Carbon Dioxide

While the principal purpose of this study is blood oxygenation, CO_2_ elimination is also an important consideration.

The outlet partial pressure of CO_2_ was estimated by performing a CO_2_ mass balance using pCO_2_ and HCO_3_^−^, together with the oxygen flow rate of 1250 ml/min.

From the pCO_2_ and HCO_3_^−^ concentrations at the inlet and outlet on each run, and treating CO_2_ binding to Hb as negligible, total CO_2_ concentrations were calculated as shown in Table 5. Using equation (2), *k*_*0*_*A* for CO_2_ was estimated for runs 1, 2, and 3 as 6.0, 6.6, and 19.4 mg·kPa^−1^·min^−1^, respectively. The 3-fold higher value for the 18N dialyser is probably due to the sensitivity of the calculation to the indirectly estimated outlet pCO_2_, and uncertainties in the bicarbonate concentrations which are calculated rather than directly measured by the ABL80 FLEX CO-OX.

The article "Toward Respiratory Support of Critically Ill COVID-19 Patients Using Repurposed Kidney Hollow Fiber Membrane Dialysers to Oxygenate the Blood" was published in 2020. Journal: J Healthc Eng.

## 4. Discussion

The minimum membrane oxygen transfer rate in the water experiments informed the decision to proceed to studies with blood.

The experiments with blood flowing at 500 ml/min yielded *k*_*0*_*A* values for oxygen which were in close agreement with the theoretically determined values and the measured value in the water study. This suggests that a Leoceed-21N HFMD would facilitate oxygen transfer rates of about 15% of the nominal 250 ml(STP)/min adult oxygen consumption rate. Using two 21N dialysers in parallel with total blood flow rates of up to 1 l/min would facilitate approximately 30% of this nominal oxygen consumption rate.

As these studies were performed at ambient pressures (85 kPa), operating at sea level and/or designing the system for increased pressure on the inlet gas may achieve an oxygen flux closer to 20% (40% with two HFMDs in parallel) of the nominal adult oxygen consumption subject to sufficient Hb in the blood.

Estimated *k*_*0*_*A* values for CO_2_ were at least an order of magnitude higher than the *k*_*0*_*A* for oxygen, suggesting that oxygenation will be rate limiting and CO_2_ elimination will be readily achieved [16]. CO_2_ elimination may even exceed its production rate, possibly requiring reduction of the fresh gas flow rate or adding CO_2_ to the fresh gas supply to limit CO_2_ losses.

## 5. Conclusions

A suitable repurposed HFMD with veno-venous access may provide a cost-effective, practical adjunct to respiratory support where ECMO is precluded.

Improvements in performance may be achievable in desperate situations by exceeding the specified maximum blood flow of 500 ml/min and increasing the gas-side pressure. However, this should be weighed against risk of damage to the unit resulting in patient harm, including air embolism.

Other considerations such as red blood cell damage, hemodynamic instability, cytokine activation, white blood cell depletion, coagulation, and bleeding are likely to be similar to those encountered in dialysis and will need to be addressed by clinicians before considering such an approach.

Dialysis pumps are costly, and presumably most are in service for renal therapy; thus, alternative low-cost pumps would be needed. However, the absence of automatic monitoring may increase risks such as undetected venous air embolisation and will require weighing the trade-offs in the face of a pandemic.

The article "Toward Respiratory Support of Critically Ill COVID-19 Patients Using Repurposed Kidney Hollow Fiber Membrane Dialysers to Oxygenate the Blood" was published in 2020. Journal: J Healthc Eng.

Further tests are essential to determine which HFMDs can be used for oxygentation and to establish the duration for which they can be operated before significant leakage occurs.

Clinical implementation would also require consideration of the placement of the venous catheters, double vs. single lumens, and the need for noncollapsible catheters under higher flow rates.

This study points to the potential for HFMD repurposing as off-label blood oxygenators in dire, resource-constrained environments. Translational research with full cooperation of regulatory authorities in various jurisdictions would be needed to assess clinical utility, feasibility, and safety prior to any consideration of clinical implementation.

## Figures and Tables

**Figure 1:** Flowsheet of the experimental setup with blood. The oxygen was passed through the dialyser via the dialysate inlet while deoxygenated blood was passed through the hollow fibers in countercurrent to the oxygen flow.

**Figure 2:** Vertically mounted Leoceed-21N HFMD showing dark deoxygenated blood entering the device at the top and bright red oxygenated blood exiting from the bottom of the device.

**Table 1:** Theoretical calculated maximum oxygen uptake per 500 ml of blood and required *k*_*0*_*A* for specified inlet conditions where the outlet is near saturation with pO_2_ of 95 mm Hg.

Inlet pO_2_ (mm Hg) (HbSat)	Max O_2_ uptake (mg/500 ml blood)	*k*_*0*_ * A* (mg·min^−1^·kPa^−1^)
45 (76%)	35.7	0.389
25 (45%)	73.4	0.787

**Table 2:** Minimum oxygen transfer rates calculated from differential dissolved oxygen concentrations between inlet and outflow water.

Water flow rate (ml/min)	Dissolved oxygen in collected water outflow (mg/l)	Calculated oxygen transfer rate (mg/min)
50	28.6	1.25
200	>32.9 (out of range)	>5.85
500	>32.9 (out of range)	>14.6

**Table 3:** Blood gas measurements at the inlet and outlet of HFMD at 500 ml/min blood flow rates over three runs. A Leoceed-21N HFMD was used for the first two runs and a Leoceed-18N was used for the third run. Measurements are reported as averages over *n* samples ±1 standard deviation uncertainty.

	pO_2_ (kPa)	pCO_2_ (kPa)	HbSat (%)
Run 1 (21N)			
Hb 10.00 ± 0.05 g/dl			
Inlet (*n* = 2)	4.55 ± 0.03	11.26 ± 0.08	37.35 ± 0.03
Outlet (*n* = 2)	15.60 ± 0.1	7.23 ± 0.05	94.70 ± 0.07

Run 2 (21N)			
Hb 10.67 ± 0.04 g/dl			
Inlet (*n* = 3)	4.87 ± 0.03	8.82 ± 0.05	43.73 ± 0.03
Outlet (*n* = 4)	9.70 ± 0.05	6.92 ± 0.04	85.75 ± 0.04

Run 3 (18N)			
Hb 11.20 ± 0.04 g/dl			
Inlet (*n* = 4)	4.20 ± 0.02	7.43 ± 0.04	42.68 ± 0.02
Outlet (*n* = 4)	10.23 ± 0.05	4.65 ± 0.02	91.08 ± 0.05

**Table 4:** Oxygen transfer rates (VO_2_) into blood for each of the three runs in ml·min^−1^. Also shown are the rounded percentages of the nominal oxygen consumption rates (VO_2,*n*_) for a typical adult of 250 ml·min^−1^ and the maximum oxygen transfer rates (VO_2,max_) calculated at the prevailing Hb for 100% HbSat at the outlet.

	VO_2_ (ml·min^−1^)	%VO_2,*n*_	%VO_2,max_
Run 1 (21N)	38.80 ± 0.03	16	91
Run 2 (21N)	29.70 ± 0.02	12	75
Run 3 (18N)	36.20 ± 0.03	15	85

The article "Toward Respiratory Support of Critically Ill COVID-19 Patients Using Repurposed Kidney Hollow Fiber Membrane Dialysers to Oxygenate the Blood" was published in 2020. Journal: J Healthc Eng.

**Table 5:** Bicarbonate concentrations, partial pressures of carbon dioxide, and total carbon dioxide flow rates at inlet and outlet of HFMD at 500 ml/min blood flow rates over three runs. As outlet gas partial pressure of carbon dioxide is approximate, the small uncertainties in measurements are not shown.

	HCO_3_^−^(mmol/l)	pCO_2_(kPa)	Total CO_2_(mmol/min)
Run 1 (21N)			
Inlet (*n* = 2)	11.62	11.26	7.10
Outlet (*n* = 2)	8.75	7.23	5.21

Run 2 (21N)			
Inlet (*n* = 3)	10.50	8.82	6.26
Outlet (*n* = 4)	8.68	6.92	5.13

Run 3 (18N)			
Inlet (*n* = 4)	10.03	7.43	5.87
Outlet (*n* = 4)	7.08	4.65	4.07

## Data Availability

Readers interested in obtaining the raw data in Excel format should send an e-mail request to the corresponding author.
